# Hub Gene Screening Associated with Early Glaucoma: An Integrated Bioinformatics Analysis

**DOI:** 10.1155/2022/8030243

**Published:** 2022-07-15

**Authors:** Rui Tian, Fuqiang Li, Songtian Che, Meijiao Song, Lu Liu, Rong Guo, Zhuoya Li, Xiaomin Hu, Hui Zhang

**Affiliations:** Department of Ophthalmology, The Second Hospital of Jilin University, Changchun, 130041 Jilin Province, China

## Abstract

**Background:**

Primary open-angle glaucoma (POAG) is the most common type of glaucoma. The potential influence of some DEGs on the progression of POAG was still incomplete. In this study, we integrated transcriptome data with clinical data to investigate the relationship between them in POAG patients.

**Methods:**

The gene expression profile (GSE27276) from Gene Expression Omnibus (GEO) was used to identify DEGs. The LIMMA package of R was used to identify the DEGs (Diboun et al., 2006). The adjusted *P* values (adj *P* value) were calculated instead to avoid the appearance of false-positive results. Genes with |log_2_ fold change (FC)| larger than 1 and adj *P* value < 0.01 were taken as DEGs between PH and PC samples. GO (Gene Ontology) function and KEGG (Kyoto Encyclopedia of Genes and Genomes) pathway enrichment analyses of the DEGs were performed. Protein-protein interactions (PPIs) of the DEGs were constructed.

**Results:**

A total of 182 DEGs were identified through our analysis, of which 119 genes were upregulated and 63 genes were downregulated. GO enrichment analysis illustrated that these DEGs were mostly enriched into haptoglobin binding, antioxidant activity, and organic acid binding. KEGG enrichment analysis illustrated that these DEGs were mostly enriched into *Staphylococcus aureus* infection. The most significant module was identified by MCODE consists of 8 DEGs, and BCL11A is the seeded gene. The second most significant module consists of 5 DEGs, and IL1RN is the seeded gene.

**Conclusion:**

Our results demonstrate the potential influence of some DEGs on the progression of POAG, providing a comprehensive bioinformatics analysis of the pathogenesis, which may contribute to future investigation into the molecular mechanisms and biomarkers.

## 1. Introduction

Primary open-angle glaucoma (POAG) is the most common type of glaucoma, accounting for 60%-70% of all glaucoma, which usually affects both eyes but is not necessarily symmetrical [1]. The morbidity of POAG increased fast and threatened the health and life of the population with population growth and aging [2, 3]. Many different abnormalities have been noted on histopathological examination of the drainage angle in patients with POAG [4]. These include narrowed intertrabecular spaces, thickened basement membranes, fused trabecular beams, reduction in trabecular endothelial cells, reduction in actin filaments, narrowing of collector channels, foreign material accumulation, scleral spur thickening, and closure of Schlemm's canal. POAG patients often find themselves with this disease when it has entered the middle and late stage of the disease, so if early detection and treatment can be achieved, the retina and optic nerve can be protected to a large extent, and the existence of effective vision of patients can be prolonged [5]. Visual loss from glaucoma is irreversible, and therefore, prevention is a key strategy to preventing morbidity from this condition.

Its pathogenesis is often related to genetic factors [6, 7]. At present, it is mainly believed that some structural changes in outflow channel of the aqueous humor caused by some factors could result in unobstructed outflow of the aqueous humor and increase of intraocular pressure, but there is basically no stenosis or obstruction in the structure of the atrial angle [8]. Intraocular pressure (IOP) is considered the most important risk factor for the development of POAG and remains the only known modifiable risk factor. Population studies have shown increased prevalence of glaucoma with increasing IOP [9]. The prevalence of POAG increases with age, even after compensating for the association between age and IOP [10]. Several studies have shown POAG to be more prevalent in people of African-Caribbean descent compared with Caucasians. Not only is POAG more prevalent in black race, its onset is earlier, and disease progression has been shown to be faster and more refractory to treatment [11]. Myopia has also been shown to be a risk factor for POAG in several studies [12].

POAG is treated with medication of first choice, namely, eye drops. Drugs that reduce the generation of aqueous humorous fluid and accelerate the outflow of aqueous humorous fluid can be selected [13, 14]. If a combination of drugs does not achieve the desired IOP, a combination formulation may be used. If drugs do not work, selective laser trabeculoplasty is an option [15]. Glaucoma surgery is the last option if the visual field progression cannot be suppressed by drugs or lasers. No matter drugs, laser, surgical treatment are to make the IOP drop to the visual field injury no longer progress level [16]. According to the etiology and inducement of POAG, the key preventive measure is to regularly monitor intraocular pressure, maintain a good attitude, and pay attention to systemic diseases [17, 18]. POAG has a genetic tendency and is generally considered to be polygenic [19]. Therefore, the family history of primary open-angle glaucoma is the most dangerous factor. People with family genetic history should go to the hospital in time for early screening of POAG.

In the present study, the differential expression of critical genes plays a key role in the mechanism of common development of the POAG and will affect therapy as well as the efficacy of medicine. Recent genome-wide studies have identified lots of novel loci associated with POAG. For example, the mutations myocilin (MYOC), optineurin (OPTN), and TANK-binding kinase 1 (TBK1) may cause POAG that is inherited as a Mendelian trait. The relationship between differentially expressed genes (DEGs) and the progression of POAG still demanded to be explained. The sharing of transcriptome data and the development of new bioinformatics analysis tools have enabled us to integrate transcriptome data with clinical data to investigate the relationship between them. This can help us understand the development of POAG from both perspectives and provide a new perspective for the prevention and treatment of the disease.

## 2. Material and Methods

### 2.1. Data

The gene expression profiles (GSE27276), which are composed of 13 controls and 15 primary open-angle glaucoma (POAG) cases, were downloaded from the Gene Expression Omnibus (GEO) database (https://www.ncbi.nlm.nih.gov/geo/) and exploited as discovery datasets to identify differentially expressed genes (DEGs). This study compared genome-wide expression profiles of individuals with and without POAG.

Of these cases, six controls and one POAG cases had the expression performed from both left and right eyes. One technical replicate was done between two cases.

### 2.2. Identification of DEGs

The LIMMA package of R was used to identify the DEGs [20]. The adjusted *P* values (adj *P* value) were calculated instead to avoid the appearance of false-positive results. Genes with |log_2_ fold change (FC)| larger than 1 and adj *P* value < 0.01 were taken as DEGs between PH and PC samples. The relevant immune genes were searched in IMMPORT (https://www.immport.org/resources) to find potential immunotherapy targets.

### 2.3. GO and KEGG Enrichment Analyses

GO (Gene Ontology) function and KEGG (Kyoto Encyclopedia of Genes and Genomes) pathway enrichment analyses of the DEGs were performed using clusterProfiler and pathview packages of R, which are designed for automating the process of biological-term classification and the enrichment analysis of gene clusters [21].

### 2.4. PPI Network Construction

Protein-protein interactions (PPIs) of the DEGs were constructed based on the Search Tool for the Retrieval of Interacting Genes (STRING; http://string.embl.de/) with the confidence score ≥ 0.9 [22]. Subsequently, the PPI network was visualized by means of Cytoscape software (version 3.5.1). Furthermore, the plugin of Molecular Complex Detection (MCODE) [23] in Cytoscape software was applied to explore the significant modules in the PPI network with default settings.

### 2.5. Statistical Analysis

Statistical calculations were carried out using SPSS statistical software (SPSS Inc., USA). For multiple comparisons, data were analyzed via analysis of variance (ANOVA) with the Tukey-Kramer Multiple Comparisons Test. *P* values < 0.05 were considered significant.

## 3. Results

### 3.1. Differentially Expressed Genes (DEGs)

The gene expression profiles (GSE27276) were used to identify DEGs, which are composed of 13 controls and 15 primary open-angle glaucoma (POAG) cases. A total of 182 DEGs were identified through our analysis, of which 119 genes were upregulated and 63 genes were downregulated (Figures 1 and 2). Of those 182 DEGs, 36 DEGs were identified as immune-related genes (Table 1). Their functions can be classified as antigen processing and presentation, antimicrobials, BCR signaling pathway, cytokines, cytokine receptors, interleukins, interleukin receptor, natural killer cell cytotoxicity, TCR signaling pathway, TGFb family member, and TNF family member receptors. Of the 36 immune-related genes, 22 DEGs were upregulated, including CHP2, CSF3, DEFB1, FABP5, FAM3B, FAM3D, GDF15, IL1RN, IL20RB, LCN2, MASP1, MTNR1A, NAMPT, S100A11, S100A12, S100A14, S100A2, S100A8, S100A9, SAA2, SERPINA3, and SLPI. Of the 36 immune-related genes, 14 DEGs were downregulated, including CCN2, CD74, CLEC11A, GPHA2, GRP, HLA-DMB, HLA-DPA1, MCHR1, OGN, PTGDS, TNFRSF25, TPM2, TYROBP, and VIM.

### 3.2. Functional Enrichment Analysis of DEGs

GO enrichment analysis illustrated that these DEGs were enriched in several terms (Figure 3), including haptoglobin binding, antioxidant activity, organic acid binding, oxygen carrier activity, peroxidase activity, oxidoreductase activity, calcium-dependent protein binding, MAP kinase phosphatase activity, fatty acid binding, oxygen binding, protein tyrosine/serine/threonine phosphatase activity, protein tyrosine/threonine phosphatase activity, RAGE receptor binding, insulin-like growth factor binding, extracellular matrix structural constituent, MAP kinase tyrosine/serine/threonine phosphatase activity, long-chain fatty acid binding, intermediate filament binding, molecular carrier activity, monocarboxylic acid binding, protein serine phosphatase activity, protein threonine phosphatase activity, structural constituent of muscle, serine-type endopeptidase activity, extracellular matrix structural constituent conferring compression resistance, growth factor binding, serine-type peptidase activity, serine hydrolase activity, protein serine/threonine phosphatase activity, and protein tyrosine phosphatase activity. KEGG enrichment analysis illustrated that these DEGs were enriched in several pathways (Figure 4). The top 10 most enriched pathways were *Staphylococcus aureus* infection, estrogen signaling pathway, tyrosine metabolism, IL-17 signaling pathway, malaria, toxoplasmosis, African trypanosomiasis, mineral absorption, phenylalanine metabolism, and histidine metabolism.

### 3.3. Protein-Protein Interaction Network

STRING was used to construct the PPI network, and the most significant modules in the PPI network were identified in Cytoscape software. The regulatory network is complex (Figure 5), and the top 5 DEGs with the highest degrees are LCN2, HP, KRT19, CDH2, and KRT5 (Figure 6). The most significant module was identified by MCODE with 8 nodes and 54 edges (Table 2). The module consists of 8 DEGs, including HP, HBG2, HBD, HBB, HBG1, HBA1, HBA2, and BCL11A. Of the 8 DEGs, BCL11A is the seeded gene. The average degree of the 8 DEGs is 6.75 and the average score is 5.84. They are enriched into two KEGG pathways, including African trypanosomiasis and malaria. The second most significant module was identified by MCODE with 5 nodes and 20 edges (Table 3). This module consists of 5 DEGs, including IL1RN, LCN2, S100A8, S100A12, and S100A9. Of the 5 DEGs, IL1RN is the seeded gene. The average degree of the 5 DEGs is 4, and the average score is 3.78. They are enriched into two KEGG pathways, including IL-17 signaling pathway and cytokine-cytokine receptor interaction.

## 4. Discussion

In the present study, the DEGs between controls and primary open-angle glaucoma (POAG) patients were explored. A total of 182 DEGs were identified through our analysis, of which 119 genes were upregulated and 63 genes were downregulated. Of the 36 immune-related genes, 22 DEGs were upregulated and 14 DEGs were downregulated. Their functions can be classified as antigen processing and presentation, antimicrobials, BCR signaling pathway, cytokines, cytokine receptors, interleukins, interleukin receptor, natural killer cell cytotoxicity, TCR signaling pathway, TGFb family member, and TNF family member receptors. GO enrichment analysis illustrated that these 182 DEGs were mostly enriched into haptoglobin binding, antioxidant activity, and organic acid binding. KEGG enrichment analysis illustrated that these 182 DEGs were mostly enriched into *Staphylococcus aureus* infection. Haptoglobin is an acute phase reactive protein [24]. Antioxidant activity is usually by preventing the diffusion stage of oxidation chain reactions [25]. This study is meaningful since transcriptome data was integrated to investigate the potential pathogenesis of DEGs between controls and primary open-angle glaucoma (POAG) patients. This study provides a reference for understanding the pathogenesis value of DEGs and formulating reasonable clinical diagnosis and treatment.

The top 5 DEGs with the highest degrees in the protein-protein network are LCN2, HP, KRT19, CDH2, and KRT5. The gene LCN2 encodes a protein that belongs to the lipocalin family. Members of this family transport small hydrophobic molecules such as lipids, steroid hormones, and retinoids [26]. The gene HP encodes a preproprotein, which is processed to yield both alpha and beta chains, which subsequently combine as a tetramer to produce haptoglobin [27]. The protein encoded by the gene KRT19 is a member of the keratin family. The keratins are intermediate filament proteins responsible for the structural integrity of epithelial cells and are subdivided into cytokeratins and hair keratins [28]. The gene CDH2 encodes a classical cadherin and member of the cadherin superfamily. Alternative splicing results in multiple transcript variants, at least one of which encodes a preproprotein proteolytically processed to generate a calcium-dependent cell adhesion molecule and glycoprotein [29]. The protein encoded by this gene KRT5 is a member of the keratin gene family. The type II cytokeratins consist of basic or neutral proteins which are arranged in pairs of heterotypic keratin chains coexpressed during differentiation of simple and stratified epithelial tissues [30].

The most significant module was identified by MCODE with 8 nodes and 54 edges. This module consists of 8 DEGs, including HP, HBG2, HBD, HBB, HBG1, HBA1, HBA2, and BCL11A. Of the 8 DEGs, BCL11A is the seeded gene. This gene BCL11A encodes a C2H2 type zinc-finger protein by its similarity to the mouse Bcl11a/Evi9 protein [31]. The corresponding mouse gene is a common site of retroviral integration in myeloid leukemia and may function as a leukemia disease gene, in part, through its interaction with BCL6. During hematopoietic cell differentiation, this gene is downregulated. It is possibly involved in lymphoma pathogenesis since translocations associated with B cell malignancies also deregulate its expression [32]. The second most significant module was identified by MCODE with 5 nodes and 20 edges. This module consists of 5 DEGs, including IL1RN, LCN2, S100A8, S100A12, and S100A9. Of the 5 DEGs, IL1RN is the seeded gene. The protein encoded by this gene IL1RN is a member of the interleukin 1 cytokine family. This protein inhibits the activities of interleukin 1, alpha (IL1A), and interleukin 1, beta (IL1B), and modulates a variety of interleukin 1-related immune and inflammatory responses, particularly in the acute phase of infection and inflammation [33, 34].

Some limitations should be acknowledged. First, only one dataset was included in the analysis, without considering the impact of population heterogeneity in different countries on the results. Second, the lack of verifiable datasets in this study limits the extrapolation of research results. Third, this study is only for the reanalysis of existing data and lacks the support and verification of experimental data. In conclusion, our results provide a comprehensive bioinformatics analysis between controls and POAG patients, which could contribute to the understanding of the development of POAG and prevention and treatment of the disease.

## 5. Conclusion

This study demonstrated the potential influence of some DEGs on the progression of POAG, providing a comprehensive bioinformatics analysis of the pathogenesis, which may contribute to future investigation into the molecular mechanisms and biomarkers.

## Figures and Tables

**Figure 1:** Volcano plots of DEGs in GSE27276.

**Figure 2:** Heatmap plots of DEGs in GSE27276.

**Figure 3:** The enriched GO terms of DEGs in GSE27276.

**Figure 4:** The enriched KEGG pathways of DEGs in GSE27276.

**Figure 5:** Protein-protein interaction network of DEGs in GSE27276.

**Figure 6:** The top 30 DEGs with the highest degree in the protein-protein interaction network.

**Table 1:** Immune-related DEGs in GSE27276.

Symbol	ID	Name	Synonyms	Chromosome	Category
CCN2	1490	Cellular communication network factor 2	CTGF|HCS24|IGFBP8|NOV2	6	Cytokines
CD74	972	CD74 molecule	DHLAG|HLADG|II|Ia-GAMMA|p33	5	Antigen_processing_and_presentation
CHP2	63928	Calcineurin-like EF-hand protein 2	—	16	BCRSignalingPathway, NaturalKiller_cell_cytotoxicity, TCRsignalingPathway
CLEC11A	6320	C-type lectin domain-containing 11A	CLECSF3|LSLCL|P47|SCGF	19	Cytokines
CSF3	1440	Colony-stimulating factor 3	C17orf33|CSF3OS|GCSF	17	Cytokines
DEFB1	1672	Defensin beta 1	BD1|DEFB-1|DEFB101|HBD1	8	Antimicrobials, chemokines, cytokines
FABP5	2171	Fatty acid-binding protein 5	E-FABP|EFABP|KFABP|PA-FABP|PAFABP	8	Antimicrobials
FAM3B	54097	FAM3 metabolism regulating signaling molecule B	2-21|C21orf11|C21orf76|ORF9|PANDER|PRED44	21	Cytokines
FAM3D	131177	FAM3 metabolism regulating signaling molecule D	EF7|OIT1	3	Cytokines
GDF15	9518	Growth differentiation factor 15	GDF-15|MIC-1|MIC1|NAG-1|PDF|PLAB|PTGFB	19	Antimicrobials, cytokines, TGFb_family_member
GPHA2	170589	Glycoprotein hormone subunit alpha 2	A2|GPA2|ZSIG51	11	Cytokines
GRP	2922	Gastrin-releasing peptide	BN|GRP-10|preproGRP|proGRP	18	Cytokines
HLA-DMB	3109	Major histocompatibility complex, class II, DM beta	D6S221E|RING7	6	Antigen_processing_and_presentation
HLA-DPA1	3113	Major histocompatibility complex, class II, DP alpha 1	DP(W3)|DP(W4)|DPA1|HLA-DP1A|HLA-DPB1|HLADP|HLASB|PLT1	6	Antigen_processing_and_presentation
IL1RN	3557	Interleukin 1 receptor antagonist	DIRA|ICIL-1RA|IL-1RN|IL-1ra|IL-1ra3|IL1F3|IL1RA|IRAP|MVCD4	2	Cytokines, interleukins
IL20RB	53833	Interleukin 20 receptor subunit beta	DIRS1|FNDC6|IL-20R2	3	Cytokine_receptors, interleukins_receptor
LCN2	3934	Lipocalin 2	24p3|MSFI|NGAL|p25	9	Antimicrobials
MASP1	5648	Mannan-binding lectin serine peptidase 1	3MC1|CRARF|CRARF1|MAP1|MASP|MASP3|MAp44|PRSS5|RaRF	3	Antimicrobials
MCHR1	2847	Melanin-concentrating hormone receptor 1	GPR24|MCH-1R|MCH1R|SLC-1|SLC1	22	Cytokine_receptors
MTNR1A	4543	Melatonin receptor 1A	MEL-1A-R|MT1	4	Cytokine_receptors
NAMPT	10135	Nicotinamide phosphoribosyltransferase	1110035O14Rik|PBEF|PBEF1|VF|VISFATIN	7	Cytokines
OGN	4969	Osteoglycin	OG|OIF|SLRR3A	9	Cytokines
PTGDS	5730	Prostaglandin D2 synthase	L-PGDS|LPGDS|PDS|PGD2|PGDS|PGDS2	9	Antimicrobials, cytokine_receptors
S100A11	6282	S100 calcium-binding protein A11	HEL-S-43|MLN70|S100C	1	Antimicrobials
S100A12	6283	S100 calcium-binding protein A12	CAAF1|CAGC|CGRP|ENRAGE|MRP-6|MRP6|p6	1	Antimicrobials
S100A14	57402	S100 calcium-binding protein A14	BCMP84|S100A15	1	Antimicrobials
S100A2	6273	S100 calcium-binding protein A2	CAN19|S100L	1	Antimicrobials
S100A8	6279	S100 calcium-binding protein A8	60B8AG|CAGA|CFAG|CGLA|CP-10|L1Ag|MA387|MIF|MRP8|NIF|P8	1	Antimicrobials
S100A9	6280	S100 calcium-binding protein A9	60B8AG|CAGB|CFAG|CGLB|L1AG|LIAG|MAC387|MIF|MRP14|NIF|P14	1	Antimicrobials
SAA2	6289	Serum amyloid A2	SAA|SAA1	11	Chemokines, cytokines
SERPINA3	12	Serpin family A member 3	AACT|ACT|GIG24|GIG25	14	Antimicrobials
SLPI	6590	Secretory leukocyte peptidase inhibitor	ALK1|ALP|BLPI|HUSI|HUSI-I|MPI|WAP4|WFDC4	20	Antimicrobials
TNFRSF25	8718	TNF receptor superfamily member 25	APO-3|DDR3|DR3|GEF720|LARD|PLEKHG5|TNFRSF12|TR3|TRAMP|WSL-1|WSL-LR	1	Cytokine_receptors, TNF_family_members_receptors
TPM2	7169	Tropomyosin 2	AMCD1|DA1|DA2B|DA2B4|HEL-S-273|NEM4|TMSB	9	Antimicrobials
TYROBP	7305	Transmembrane immune signaling adaptor TYROBP	DAP12|KARAP|PLOSL|PLOSL1	19	NaturalKiller_cell_cytotoxicity
VIM	7431	Vimentin	—	10	Antimicrobials

**Table 2:** The most significant module in the PPI network.

Gene	Node status	Score
HP	Clustered	6
HBG2	Clustered	5.785714
HBD	Clustered	5.785714
HBB	Clustered	5.785714
HBG1	Clustered	5.785714
HBA1	Clustered	5.785714
HBA2	Clustered	5.785714
BCL11A	Seed	6

**Table 3:** The second most significant module in the PPI network.

Gene	Node status	Score
IL1RN	Seed	4
LCN2	Clustered	3.733333
S100A8	Clustered	3.733333
S100A12	Clustered	3.733333
S100A9	Clustered	3.733333

## Data Availability

The data used to support this study is available from the corresponding author upon request.
